# Exploring the Thoracolumbar Interfascial Plane (TLIP) Block as a Novel Approach for Improved Pain Management After Spine Surgery: A Comparative Review

**DOI:** 10.7759/cureus.59531

**Published:** 2024-05-02

**Authors:** Sweta J Gajapure, Vivek Chakole

**Affiliations:** 1 Anesthesiology, Jawaharlal Nehru Medical College, Datta Meghe Institute of Higher Education and Research, Wardha, IND

**Keywords:** analgesia, thoracolumbar junction, regional anesthesia, postoperative pain management, spine surgery, tlip block

## Abstract

Postoperative pain management following spine surgery remains a significant challenge, often requiring multimodal approaches to achieve adequate analgesia while minimizing side effects. The thoracolumbar interfascial plane (TLIP) block has emerged as a novel regional anesthesia technique for addressing this issue. By targeting the interfascial plane between the erector spinae and quadratus lumborum muscles at the thoracolumbar junction, the TLIP block aims to provide targeted analgesia to the surgical site while reducing systemic opioid requirements. This review explores the anatomy, technique, mechanism of action, and clinical evidence supporting the TLIP block for post-spine surgery pain management. Additionally, it compares the TLIP block with traditional pain management approaches and discusses its implications for clinical practice and future research. Overall, the TLIP block shows promise as an effective and potentially safer alternative for post-spine surgery pain management, potentially improving patient outcomes and enhancing recovery. Further research is warranted to optimize its utilization and comprehensively evaluate its long-term effects.

## Introduction and background

Spine surgery, while often necessary for various conditions such as herniated discs, spinal stenosis, or deformities like scoliosis, is frequently accompanied by significant postoperative pain. This pain can hinder patient recovery, impair mobility, delay rehabilitation, and affect the overall quality of life [1]. Conventional pain management strategies, such as systemic opioids, nonsteroidal anti-inflammatory drugs (NSAIDs), and epidural analgesia, may be effective but are not without limitations, including side effects and potential risks of complications [2]. The thoracolumbar interfascial plane (TLIP) block is a novel regional anesthesia technique that has gained attention for its potential to provide effective analgesia following spine surgery [3]. This technique involves the precise deposition of local anesthetic within the interfascial plane between the erector spinae and quadratus lumborum muscles at the thoracolumbar junction. By targeting this specific anatomical region, the TLIP block aims to interrupt nociceptive signals from the surgical site, thereby mitigating postoperative pain [4].

The primary objective of this review is to evaluate the efficacy of the TLIP block as a modality for managing post-spine surgery pain. Through a comprehensive examination of available literature, including randomized controlled trials (RCTs), comparative studies, and meta-analyses, this review provides insights into the clinical effectiveness, safety profile, and potential advantages of the TLIP block compared to traditional pain management approaches. Ultimately, the aim is to contribute to a better understanding of the TLIP block and its role in optimizing postoperative pain control for patients undergoing spine surgery.

## Review

Mechanism of action

Local Anesthetic Distribution and Nerve Involvement

The TLIP block is a regional anesthesia technique that specifically targets the dorsal rami of the thoracolumbar nerves. This is achieved by injecting a local anesthetic into the fascial plane situated between the multifidus and longissimus muscles, typically around the level of the third lumbar vertebra (L3) [5,6]. Research indicates that this method offers prolonged postoperative analgesia while notably reducing the need for opioids, all while minimizing the risks commonly associated with neuraxial and plexus blocks [6]. Studies have demonstrated the efficacy of the TLIP block in alleviating postoperative pain at rest and during movement within the initial 24-hour period following surgery, with its peak effectiveness observed around the two-hour mark postoperatively [5]. The TLIP block has exhibited superior results in reducing pain scores and total analgesic consumption compared to local anesthetics' wound infiltration. Notably, the TLIP block has been associated with a significant decrease in analgesic requirement compared to scenarios involving no or sham block and wound infiltration [5]. However, it is worth noting that while the TLIP block has shown a reduction in pain scores at eight hours postoperatively when compared to wound infiltration, no statistically significant difference was observed at other time points [5]. Furthermore, the TLIP block has been found effective in managing postoperative pain following lumbar discectomy. Studies have reported a notable decrease in the visual analog scale for pain and reduced cumulative morphine consumption in patients who received the TLIP block compared to those in the control group [7]. Additionally, the TLIP block group exhibited a significant decrease in nausea and a lower incidence of sedation than the control group [7]. These findings collectively suggest the potential of the TLIP block as a valuable tool in post-spine surgery pain management, offering both effective pain relief and improved patient outcomes.

Blocking Nociceptive Signals From the Surgical Site

Blocking nociceptive signals from the surgical site is a pivotal element in postoperative pain management for spine surgeries. The TLIP block precisely targets the sensory innervation of the thoracolumbar region by administering local anesthetics into the fascial plane situated between specific muscles, such as the multifidus and longissimus paraspinal muscles or the longissimus and iliocostalis muscles [5,8]. This focused approach toward the dorsal rami of the thoracolumbar nerves effectively diminishes postoperative pain at rest and during movement, culminating in enhanced pain control for up to 24 hours following surgery [3,5]. Studies have underscored the significant reduction in postoperative opioid consumption and pain scores achieved with the TLIP blocks compared to reliance solely on general anesthesia, thus positioning them as a valuable alternative to systemic opioids for post-spinal surgery pain management [5]. Moreover, the TLIP blocks have exhibited a decrease in overall analgesic usage and the occurrence of postoperative nausea and vomiting (PONV), further accentuating their efficacy in intercepting nociceptive signals from the surgical site and fostering patient comfort and favorable outcomes [3].

Modulation of Sympathetic Activity

The autonomic nervous system (ANS) profoundly influences the heart's structural integrity and electrical conductivity. Dysregulated activation of the sympathetic nervous system can provoke heterogeneous changes with arrhythmogenic potential, contributing to the onset of atrial tachyarrhythmias and atrial fibrillation (AF). Targeting autonomic activity, particularly by attenuating sympathetic outflow, has demonstrated efficacy in reducing the occurrence of spontaneous or induced atrial tachyarrhythmias and AF, suggesting the potential utility of such interventions in AF management [9]. The ANS, with particular emphasis on the sympathetic nervous system, plays a pivotal role in initiating and perpetuating AF. Modulating ANS function represents a vital therapeutic strategy for enhancing AF management in specific patient populations. Potential therapeutic modalities encompass pharmacological inhibition utilizing central and peripheral sympatholytic agents and sympathetic neuromodulation techniques [9]. Additionally, the vestibular system has been identified as a regulator of sympathetic nerve activity (MSNA) in humans' muscles and skin. Vestibular inputs modulate MSNA, exhibiting a stronger temporal coupling during inspiratory phases of respiration and competing with baroreceptor inputs. Studies have elucidated the vestibulosympathetic reflex, with neurons in the rostral ventrolateral medulla of felines exhibiting responses to natural vestibular stimulation. Notably, vestibular stimulation in humans elicits sympathetic responses, with caloric stimulation enhancing sympathetic outflow to the skin and natural stimulation of horizontal semicircular canals augmenting sympathetic outflow to the muscle [10]. Furthermore, the respiratory modulation of sympathetic activity has been investigated, revealing a correlation between sympathetic activity and respiratory phases, with the brainstem playing a central role in this modulation. Respiratory activity influences sympathetic activity: the brainstem's involvement is instrumental in orchestrating this modulation [11].

Clinical evidence supporting the TLIP block

RCTs Assessing the TLIP Block Efficacy

The TLIP block stands out as a pioneering regional anesthesia technique, demonstrating noteworthy effectiveness in alleviating postoperative pain intensity, diminishing opioid consumption, mitigating side effects, and curbing requests for rescue analgesia following spinal surgeries [3,5,6,12]. A comprehensive meta-analysis encompassing 17 RCTs revealed that the TLIP blocks notably reduced pain scores at rest and during movement for up to 24 hours postoperatively. Additionally, the TLIP blocks exhibited a substantial decrease in total analgesic consumption and a reduced incidence of PONV, specifically after lumbar spinal surgeries [3]. In direct comparison to wound infiltration, the TLIP blocks proved superior in terms of opioid consumption, while postoperative pain intensity at rest remained comparable between the TLIP block and wound infiltration techniques [3,12]. Furthermore, a meta-analysis of nine studies corroborated these findings, showcasing a significant reduction in pain scores and total analgesic consumption with the TLIP blocks. Interestingly, pain scores between the TLIP blocks and wound infiltration were identical, albeit with a noteworthy decrease in total analgesic consumption with the TLIP blocks [13]. However, it is crucial to exercise caution in interpreting these results due to the scarcity of evidence regarding the TLIP block's efficacy compared to wound infiltration of local anesthetics. The quality of primary studies ranges from low to moderate, and significant heterogeneity warrants careful consideration when evaluating the findings [13]. Despite these limitations, the accumulating evidence underscores the potential of the TLIP blocks as a promising approach to optimizing postoperative pain management strategies following spinal surgeries.

Comparative Studies Against Conventional Pain Management Techniques

The TLIP block represents a recent advancement in regional anesthesia techniques, demonstrating notable efficacy in mitigating postoperative pain intensity, reducing opioid consumption, minimizing side effects, and diminishing requests for rescue analgesia following spinal surgery [14,15]. A comprehensive meta-analysis comprising 17 RCTs revealed that the TLIP blocks significantly decreased pain scores at rest and during movement for up to 24 hours postoperatively. Additionally, the TLIP blocks exhibited a marked reduction in total analgesic consumption and a lowered incidence of PONV, specifically after lumbar spinal surgeries [16]. Compared to wound infiltration, the TLIP blocks were found to be superior in terms of opioid consumption. At the same time, the postoperative pain intensity at rest remained comparable between the TLIP block and wound infiltration techniques [14,15]. Moreover, a meta-analysis of nine studies echoed these findings, indicating a significant reduction in pain scores and total analgesic consumption with the TLIP blocks. Interestingly, pain scores between the TLIP blocks and wound infiltration were identical, albeit with a substantial decrease in total analgesic consumption with the TLIP blocks [3]. Nevertheless, it is imperative to approach these findings with caution due to the scarcity of evidence regarding the TLIP block's efficacy compared to wound infiltration of local anesthetics. The quality of primary studies ranges from low to moderate, and significant heterogeneity among them necessitates careful interpretation of the results [3]. Despite these limitations, the accumulating evidence underscores the potential of the TLIP blocks as a promising strategy in optimizing postoperative pain management strategies following spinal surgeries.

Comparative analysis with other regional anesthesia techniques

Comparing the TLIP Block With Epidural Analgesia

When comparing the TLIP block with epidural analgesia, the TLIP block emerges as a promising option for postoperative pain management following spine surgery. Studies have consistently demonstrated the effectiveness of the TLIP blocks in reducing postoperative pain intensity, opioid consumption, and the incidence of PONV when compared to standard care without blocks and wound infiltration techniques [17-19]. The TLIP blocks have shown significant reductions in opioid consumption during the initial 24 hours post-surgery, along with decreased postoperative pain intensity at rest and during movement, ultimately resulting in decreased reliance on rescue analgesia [18,19]. On the other hand, epidural analgesia represents a well-established method for pain control following spine surgery. While effective in providing pain relief, epidural analgesia is associated with potential risks such as hypotension, urinary retention, and the formation of epidural hematomas. In contrast, the TLIP blocks offer a regional anesthesia technique specifically targeting the dorsal rami of the thoracolumbar nerves, providing an alternative to systemic opioids and potentially reducing the risk of adverse events commonly associated with epidural analgesia. The TLIP blocks present a promising avenue for postoperative pain management after spine surgery, offering effective pain relief while potentially mitigating the risks associated with epidural analgesia. Further research and clinical experience will continue to refine our understanding and utilization of the TLIP blocks in optimizing patient care and outcomes following spinal procedures. Table 1 compares the TLIP block with other blocks.

**Table 1:** Comparing the TLIP block with other blocks

Feature	TLIP Block	Epidural Analgesia	Paravertebral Block
Anatomical target	Between the erector spinae and quadratus lumborum muscles at the thoracolumbar junction.	Epidural space around the spinal cord.	Paravertebral space is adjacent to the vertebral column.
Indications	Post-spine surgery pain management.	Postoperative pain management in abdominal, thoracic, and lower limb surgeries.	Thoracic, abdominal surgery, and some types of spine surgery.
Technique	Ultrasound-guided needle placement.	Catheter placement guided by anatomical landmarks, possibly assisted by fluoroscopy.	Ultrasound-guided or landmark-based needle insertion.
Analgesia coverage	Localized to the thoracolumbar region.	Broad coverage, depending on catheter placement level, can be segmental.	Primarily unilateral, segmental coverage adjacent to the site of the block.
Complications	Nerve injury, bleeding, local anesthetic toxicity, infection.	Hypotension, urinary retention, infection, epidural hematoma, dural puncture headache.	Pneumothorax, nerve injury, local anesthetic toxicity, infection.
Advantages	Minimizes systemic opioid use and fewer systemic side effects.	Extensive pain control, continuous infusion option.	Unilateral block reduces systemic effects, which is good for unilateral surgical procedures.
Disadvantages	Limited to specific surgical sites, newer techniques with less long-term data.	Invasive risk of severe complications like epidural hematoma and motor block.	The risk of pneumothorax is limited to procedures on one side of the body.
Patient mobility	Generally, allows greater mobility post-procedure.	Depending on the local anesthetic used, it can limit mobility due to motor block.	Generally, does not impair mobility unless motor nerves are affected.

Comparing the TLIP Block With a Paravertebral Block

When comparing the TLIP block with a paravertebral block (PVB), evidence suggests that PVB may offer superior pain relief following thoracoscopic surgery [18]. One study revealed that patients receiving PVB exhibited faster ambulation than those receiving the TLIP block, and none of the patients in the PVB group experienced complete motor blockade, which was observed in all patients receiving the TLIP block [20]. However, it is worth noting that the time to first analgesic requirement and the duration of block performance were significantly prolonged in the PVB group, and patients in this group reported lower satisfaction levels than those in the TLIP block group [20]. Conversely, a meta-analysis of RCTs indicated that erector spinae plane block (ESPB) may provide superior pain relief after thoracoscopic surgery compared to PVB [21]. This analysis found that ESPB significantly reduced pain scores at 12 hours postoperatively and decreased postoperative analgesic consumption compared to PVB. However, both groups exhibited similar pain scores at 1-2 hours and 4-6 hours postoperatively, as well as comparable incidences of nausea and vomiting [21]. While PVB may offer better pain relief than the TLIP block following thoracoscopic surgery, it is associated with prolonged time to first analgesic requirement and block performance, as well as lower patient satisfaction levels. Additionally, ESPB may represent a superior alternative to PVB in terms of pain relief and postoperative analgesic consumption. Further research is warranted to elucidate the optimal regional anesthesia technique for pain management in thoracoscopic surgery settings.

Advantages and Disadvantages of the TLIP Block Over Other Techniques

The TLIP block emerges as a novel regional anesthesia technique demonstrating efficacy in providing effective postoperative pain relief following spine surgery. Compared to non-block care, the TLIP block has been shown to significantly diminish postoperative pain intensity at rest and during movement across various time points. Furthermore, it surpasses wound infiltration in reducing opioid consumption [19]. Integrating the TLIP block into a perioperative, multimodal, opioid-sparing analgesic regimen has the potential to substantially contribute to enhanced recovery times after lumbosacral spine surgery [22]. This technique functions by averting pain occurrence through its targeted action on the dorsal rami of the spinal nerves, thereby furnishing adequate analgesia even for procedures as extensive as lumbar spinal fusion surgery [22]. Notably, the TLIP block administered at the L3 vertebral level has been reported to establish an analgesic area encompassing the middle and lower back [22]. However, despite its promising efficacy, more reports need to detail the application of the TLIP block in RCTs, specifically concerning lumbosacral spine surgery [22]. In contrast to other regional anesthesia techniques, the TLIP block presents several advantages. It is less invasive than epidural anesthesia, which necessitates the placement of a catheter in the epidural space, thereby reducing the associated risks of complications such as epidural hematoma or abscess [23]. Moreover, the TLIP block provides a broader area of analgesia compared to wound infiltration with local anesthetic, which is confined to the surgical incision site [6]. Nonetheless, there are inherent drawbacks to the TLIP block. Its execution requires ultrasound guidance to ensure precise placement of the local anesthetic in the the TLIP, a resource that may not be universally available across all clinical settings [23]. Additionally, the duration of the block may be shorter compared to other regional anesthesia techniques, such as epidural anesthesia, which may necessitate the implementation of catheters for continuous infusion of local anesthetic [23].

Safety profile and complications

Incidence of Complications Associated With the TLIP Block

Based on available evidence, the incidence of complications associated with the TLIP block appears to be low. A systematic review and meta-analysis comprising 17 RCTs reported no major adverse events or complications related to the TLIP block or wound infiltration [19]. Pooled data from four studies indicated a significant reduction in the incidence of rescue analgesia requirement with the TLIP block (95% confidence interval (CI) 0.30, 0.74; p = 0.001; I2 = 0.0%) [19]. Furthermore, one study revealed that patients receiving the TLIP block experienced a lower incidence of PONV compared to those receiving wound infiltration (relative risk (RR) 95% CI 0.05, 0.852; p = 0.029) [19]. The reported incidence of an unsuccessful TLIP block was 0.8% (95% CI 0.3%, 2%) [19]. In a case report involving a cirrhotic hepatic patient with thrombocytopenia undergoing endoscopic spinal decompression with laminotomy and flavectomy of L4-L5, a modified TLIP block performed at the L3 level was found to be safe. The patient did not experience any neurological complications or bleeding attributable to the modified TLIP block [24]. While the available evidence suggests that complications associated with the TLIP block are rare, careful consideration and adherence to appropriate patient selection criteria and procedural techniques remain essential to minimize risks and ensure patient safety. Figure 1 shows complications associated with the TLIP block.

**Figure 1:** Complications associated with the TLIP block TLIP, thoracolumbar interfascial plane Image credits: Sweta J. Gajapure. Source [19,24]

Comparison of Complication Rates With Other Regional Anesthesia Methods

The TLIP block demonstrates a favorable safety profile, with various studies reporting no major adverse events or complications associated with its use [19,25]. In spine surgery patients, the TLIP block has shown clinical superiority over non-block care in terms of postoperative pain management, opioid consumption, rescue analgesia requirement, and the incidence of PONV [19]. Furthermore, the TLIP block has been found to reduce opioid consumption compared to wound infiltration while maintaining comparable postoperative pain intensity at rest [19]. These findings underscore the safety and efficacy of the TLIP block, highlighting its potential as a promising regional anesthesia technique for spine surgery. However, it is crucial to acknowledge that while the TLIP block demonstrates positive outcomes in pain management and opioid reduction, further quantitative studies are necessary to compare complication rates with other regional anesthesia methods. This will provide a comprehensive understanding of the TLIP block's safety profile relative to alternative techniques [19,25]. Continued research in this area will contribute to refining clinical practices and optimizing patient outcomes in spine surgery.

Strategies for Minimizing Risks and Managing Complications

The TLIP block represents a novel approach for enhancing pain management following spine surgery. Generally, the safety profile of the TLIP block appears favorable, with several studies reporting no complications or adverse events [19,26]. However, it is essential to acknowledge potential risks, such as the possibility of neuraxial injury and challenges associated with sonographic imaging during the TLIP block administration [19]. Adherence to proper techniques and guidelines for the TLIP block administration is imperative to mitigate risks and address potential complications. This includes utilizing ultrasound guidance to ensure precise needle placement, employing local anesthetics with safe dosages, and monitoring patients for any signs of complications, such as neurological deficits or hematoma formation [26,27]. Moreover, weighing the potential risks and benefits of the TLIP block compared to alternative pain management techniques is crucial. While the TLIP block has demonstrated significant reductions in postoperative pain intensity compared to non-block care, evidence regarding its efficacy relative to wound infiltration of local anesthetics is limited [19]. Consequently, interpretation of results should be approached cautiously due to the variability in study quality and significant heterogeneity among primary studies [19].

Clinical applications and considerations

Patient Selection Criteria for the TLIP Block

The TLIP block emerges as a novel approach for enhancing postoperative pain management following spine surgery, as evidenced by its significant reduction in postoperative pain intensity compared to non-block care at various time points [28,29]. This technique holds promise for effectively alleviating pain and reducing opioid consumption in spine surgery patients. However, further research is warranted to substantiate its long-term benefits and to compare its efficacy with alternative pain management strategies. Patient selection criteria for the TLIP block implementation typically include individuals undergoing single-level lumbar surgery, as supported by an RCT demonstrating the efficacy of the TLIP block as part of multimodal analgesia in such patients [29]. Additionally, a pilot study involving volunteers revealed that ultrasound-guided injection of local anesthetic into the fascial plane yields a reproducible area of anesthesia [28]. Nevertheless, it is essential to consider certain factors, such as the extent of the block reported in centimeters rather than dermatomes, as well as the height and body mass index (BMI) of the individuals, as these factors may influence the achieved extent of the block [28]. Figure 2 shows the patient selection criteria for the TLIP block.

**Figure 2:** Patient selection criteria for the TLIP block TLIP, thoracolumbar interfascial plane Image credits: Sweta J. Gajapure. Source [28,29]

Timing and Dosage Considerations

While the optimal timing and dosage considerations for the TLIP block in spine surgery are not explicitly stated in the available search results, the studies suggest that the TLIP block is indeed effective in reducing postoperative pain intensity at rest or during movement at various time points compared with non-block care [19,30]. A quantitative systematic review highlighted the TLIP block's efficacy in decreasing opioid consumption within the first 24 hours post-surgery compared to non-block care, with secondary outcomes including reduced postoperative pain intensity, decreased rescue analgesia requirement, and lower incidence of PONV [19]. Additionally, the TLIP block was found to be superior to wound infiltration in terms of opioid consumption, while postoperative pain intensity at rest was comparable between the TLIP block and wound infiltration [19]. Regarding dosage, some studies suggest the administration of 30 ml of 0.375% ropivacaine bilaterally into the interfascial plane between the longissimus and iliocostalis muscles [31]. However, it is important to note that the optimal dosage and timing of the TLIP block in spine surgery require further investigation to establish standardized protocols and guidelines. Continued research efforts are essential to refine our understanding of the TLIP block's efficacy and optimize its utilization in clinical practice.

Combination Therapy With Systemic Analgesics and Adjuncts

While the optimal timing and dosage considerations for the TLIP block in spine surgery are not explicitly stated in the available search results, the studies suggest that the TLIP block is indeed effective in reducing postoperative pain intensity at rest or during movement at various time points compared with non-block care [19,30]. A quantitative systematic review highlighted the TLIP block's efficacy in decreasing opioid consumption within the first 24 hours post-surgery compared to non-block care, with secondary outcomes including reduced postoperative pain intensity, decreased rescue analgesia requirement, and lower incidence of PONV [19]. Additionally, the TLIP block was found to be superior to wound infiltration in terms of opioid consumption, while postoperative pain intensity at rest was comparable between the TLIP block and wound infiltration [19]. Regarding dosage, some studies suggest the administration of 30 ml of 0.375% ropivacaine bilaterally into the interfascial plane between the longissimus and iliocostalis muscles [25]. However, it is important to note that the optimal dosage and timing of the TLIP block in spine surgery require further investigation to establish standardized protocols and guidelines. Continued research efforts are essential to refine our understanding of the TLIP block's efficacy and optimize its utilization in clinical practice.

## Conclusions

In conclusion, the TLIP block is promising for managing post-spine surgery pain. Targeting the specific anatomical region between the erector spinae and quadratus lumborum muscles, the TLIP block offers a focused approach to analgesia while potentially mitigating the systemic side effects associated with traditional pain management methods. Its precision and mechanism of action underscore its appeal as an adjunct to multimodal pain management strategies following spine surgery. Incorporating the TLIP block into standardized protocols may lead to improved postoperative recovery outcomes and reduced reliance on systemic opioids. However, further research is necessary to optimize techniques, dosing, and patient selection criteria. Comparative studies and long-term outcome assessments will definitively elucidate the role of the TLIP block. Overall, the TLIP block significantly impacts patient outcomes by enhancing pain control, satisfaction, and recovery trajectories in the post-spine surgery setting, potentially reshaping clinical practice paradigms in spinal anesthesia.
